The article "Bibliometric Analysis of the Role of Occludin in the Pathogenesis of Stroke" was published in 2024. Journal: Oxid Med Cell Longev.

# Bibliometric Analysis of the Role of Occludin in the Pathogenesis of Stroke

**DOI:** 10.1155/2024/2121733

**Published:** 2024-08-01

**Authors:** Zhanylsyn U. Urasheva, Gulnar B. Kabdrakhmanova, Aigul P. Yermagambetova, Aigerim B. Utegenova, Nazgul A. Seitmaganbetova, Ondassyn M. Aliyev, Saulesh S. Kurmangaliyeva, Nazym K. Kenzhina, Yergen Z. Kurmambayev, Alima A. Khamidulla

**Affiliations:** ^1^ Department of Neurology West Kazakhstan Marat Ospanov Medical University, Aktobe, Kazakhstan; ^2^ Department of Propaedeutics of Internal Diseases West Kazakhstan Marat Ospanov Medical University, Aktobe, Kazakhstan; ^3^ Department of Microbiology, Virology and Immunology West Kazakhstan Marat Ospanov Medical University, Aktobe, Kazakhstan; ^4^ The Course of Therapy West Kazakhstan High Medicine College, Uralsk, Kazakhstan; ^5^ Department of Internal Medicine 1 West Kazakhstan Marat Ospanov Medical University, Aktobe, Kazakhstan

## Abstract

Over the past decade, there has been a notable surge in research dedicated to unraveling the intricate role of tight junction proteins in blood–brain barrier (BBB) damage associated with ischemic stroke. This bibliometric analysis explores the expansive landscape of occludin research, a key tight junction protein, during the years 2000–2023, shedding light on the global scientific contributions, collaborations, and emerging trends in this critical area of stroke pathogenesis. China and the United States emerge as significant contributors, underscoring their prominence in advancing our understanding of tight junction proteins. Occludin, identified as a linchpin in regulating BBB integrity, proves to be a pivotal player, with implications extending to the diagnosis of hemorrhagic transformation in ischemic stroke. This study identifies occludin as a potential biomarker, offering promise for early diagnosis and paving the way for novel diagnostic strategies. The analysis highlights the necessity for a more comprehensive exploration of tight junction proteins, including occludin and claudin-5, particularly in the context of acute cerebral ischemia. The unique healthcare landscape in Kazakhstan adds urgency to the call for further scientific research in this region, emphasizing the need for tailored investigations to address specific regional challenges. This comprehensive overview not only delineates the current state of occludin research but also signals the direction for future investigations. The identified knowledge gaps and emerging trends provide a roadmap for researchers and policymakers alike, with implications for both scientific discourse and clinical practice. Moving forward, a deeper understanding of tight junction proteins, informed by the insights gleaned from this study, holds the potential to shape targeted therapeutic interventions and diagnostic strategies, ultimately contributing to advancements in global stroke care.

The article "Bibliometric Analysis of the Role of Occludin in the Pathogenesis of Stroke" was published in 2024. Journal: Oxid Med Cell Longev.

## 1. Introduction

Stroke remains a formidable global health challenge, ranking as the fifth leading cause of death and contributing to a substantial burden of disability worldwide [1]. The staggering toll of stroke is reflected in the estimated 5.5 million fatalities annually, accounting for approximately 44 million disability-adjusted life-years [2]. Recent data from 2020 reveals a worldwide prevalence of 89.13 million stroke cases, with acute ischemic stroke affecting a noteworthy 68.16 million individuals [3]. In the context of Kazakhstan, stroke emerges as the second most prevalent cause of mortality, surpassed only by cardiovascular pathology, and claims the top spot in disability rates [4]. The incidence of cerebral stroke in various regions of Kazakhstan underscores its significance, with annual rates reaching 2,373 people per million individuals, accompanied by mortality rates ranging from 398 to 720 people per million individuals [4]. Official statistics from the Ministry of Health in the Republic of Kazakhstan report over 40,000 registered cases of stroke annually, among which 5,000 succumb within the initial 10 days, and another 5,000 within 1 month after discharge to home [4].

Despite these alarming statistics, the underlying mechanisms, and molecular contributors to stroke pathology remain complex and multifaceted. Ischemic stroke, constituting 62.4% of all stroke incidents, poses a significant health threat, with diverse etiologies such as atherosclerotic lesions, cardiac emboli, and acute thrombosis in the context of other diseases [5, 6]. Following an ischemic stroke, the ensuing cerebral ischemia and reperfusion injury unleash a cascade of deleterious consequences, including oxidative stress, intracellular calcium overload, neural cell apoptosis, and compromise of the blood–brain barrier (BBB) [7].

The current gold standard for ischemic stroke treatment, recombinant tissue plasminogen activator, is hampered by a narrow treatment time window and the risk of inducing bleeding, limiting its widespread application [8]. This therapeutic approach primarily targets the disruption of the BBB and reperfusion injury, elucidating the significance of understanding BBB dynamics in stroke pathology [9, 10]. Notably, during brain tissue ischemia, the release of inflammatory factors directly damages the BBB, heightening its permeability and facilitating the infiltration of detrimental substances into brain tissue, thereby exacerbating damage to neural cells [10].

The article "Bibliometric Analysis of the Role of Occludin in the Pathogenesis of Stroke" was published in 2024. Journal: Oxid Med Cell Longev.

The BBB, a crucial component of cerebral vascular integrity, is primarily composed of brain microvascular endothelial cells lining cerebral capillaries, supported by the surrounding basement membrane, pericytes, and astrocytes [10]. The integrity of the BBB heavily relies on endothelial cells and the tight junctions between them [11]. The tight junctions between these endothelial cells, comprised of various proteins such as occludin, claudins, intracellular zonula occludens-1 (ZO-1), and junction adhesion molecules, play a pivotal role in maintaining BBB permeability and overall structural integrity [12]. Reduction in proteins like occludin and ZO-1 leads to structural alterations in tight junctions, increasing BBB permeability and resulting in the formation of cerebral edema [13]. Specifically, occludin, as a structural component of tight junctions, emerges as a key player in preserving the barrier function of the BBB [14].

Against this background, our study aims to conduct a comprehensive bibliometric analysis, which allows us to identify important scientific publications, research trends, and main directions of research in the field of studying the role of occlusion in the pathogenesis of consultation. In particular, we focused on an article on bibliometric analysis, which provides methodological approaches and examples of the use of this method in biomedical research [15]. By synthesizing existing literature and exploring the scientific landscape surrounding occludin in the context of stroke, we seek to contribute valuable insights into the molecular mechanisms underpinning BBB dysfunction and the development of ischemic stroke. Through a systematic examination of occludin-related research, we aspire to identify knowledge gaps, highlight key findings, and pave the way for future investigations aimed at advancing our understanding of stroke pathology and refining therapeutic strategies.

## 2. Materials and Methods

### 2.1. Search Results

In November 2023, Scopus was utilized to gather data for a comprehensive examination of occludin's role in BBB damage during ischemic stroke pathogenesis. The search strategy implemented aimed at inclusivity and covered various facets of the subject matter. The specific search strategy employed was “stroke” AND “blood” AND “brain” AND “barrier” AND “occludin” (title and abstract).

To ensure data accuracy and relevance, stringent inclusion criteria were applied. These criteria encompassed articles published between 2000 and 2023, articles exclusively in English, and the exclusion of review articles, proceedings, book chapters, and editorial materials. To provide a visual representation of the data extraction process, a PRISMA flowchart outlining the selection process is presented in Figure 1.

The article "Bibliometric Analysis of the Role of Occludin in the Pathogenesis of Stroke" was published in 2024. Journal: Oxid Med Cell Longev.

### 2.2. Performance Analysis

The study involved performance analysis and scientific mapping using specialized software tools. RStudio v.4.3.1, along with the bibliometric R-package, was employed for these analyses. Biblioshiny, equipped with web functionalities, was utilized for data analysis. Notably, this software operates with a single database. The Scopus was selected for its comprehensive citation information, which is instrumental in conducting meticulous bibliometric analyses and evaluating research impact. This feature is particularly valuable for conducting thorough bibliometric analysis and assessing the impact of research outputs.

### 2.3. Identification of Leading Institutions, Sources, Authors, and Collaborating Countries

The top 10 most prolific institutions and authors were ranked according to the percentage of papers they generated. Visualization techniques were employed to elucidate collaboration patterns among institutions and authors. In the context of country analysis, the proportion of articles originating from each country was employed to determine the most productive country, while the percentage of collaborative efforts involving multiple countries was assessed for the top 10 countries. A country collaboration network was constructed, mapping the relationships based on the number of publications produced by each country.

### 2.4. Keywords Frequencies Analysis

Timeline analysis was conducted to observe the temporal frequency of specific keywords over the years. A TreeMap was generated to visually represent the distribution and prominence of the top 10 most frequently occurring keywords. Additionally, thematic analysis was employed to identify the principal trends and topics within the selected articles.

## 3. Results

### 3.1. Analyzing Trends, Citations, and Collaborations

This study aimed to conduct a comprehensive examination of the role of occludin in stroke pathogenesis spanning the years 2000–2023. Bibliographic data were sourced from the Web of Science and Scopus databases, with the search period not restricted. Documents were filtered for Article and Review types, and English language preference. A meticulous review of 197 pertinent studies from 114 distinct sources was undertaken. The analysis encompassed the contributions of 1,116 authors, yielding an impressive average of 36.92 citations per document over the entire period. The earliest article dated back to 2000. Key findings elucidating the role of occludin in stroke pathogenesis, primarily derived from the most prolific papers in 2021–2022, are depicted in Figure 2. Furthermore, the annual growth rate for this research field was calculated at 12.36%, indicating a consistent increase in publications throughout the study period. The substantial research output is underscored by the inclusion of one reference and 519 unique author keywords. Notably, a quarter of the authors engaged in collaborative research, accounting for 23.86% of the total contributors.

The article "Bibliometric Analysis of the Role of Occludin in the Pathogenesis of Stroke" was published in 2024. Journal: Oxid Med Cell Longev.

### 3.2. Identifying Key Journals and Prolific Contributors

Utilizing Bradford's law, which describes the distribution of scientific articles among different journals, we identified 12 core journals that were deemed to be the top choices for researchers. According to Bradford's law, these specialized journals collectively account for a significant portion of the total number of published articles on occludin in ischemic stroke (Figure 2). Upon analyzing the publication data from these core journals, we observed that the journals “Brain Research” and “Scientific Reports” emerged as the most prolific ones, contributing a substantial seven articles, which represents approximately 3.5% of the total articles within the study period. Furthermore, we investigated the local citations received by these core journals from other articles within our dataset.

### 3.3. Journal and Author Dynamics

The most published journals on stroke and occludin have become “Brain Research” and “Scientific Reports,” which each published nine articles, which amounted to 4.57% (Figure 3). Among the authors, Zhang Y stood out with the highest number of articles (15, 5.9%), followed by Wang Y, who produced 14 articles (Figure 4).

The most often published writers on the function of occludin in the aetiology of stroke are depicted in Figure 5. Chinese researchers have made important advances in our understanding of occludin in stroke. In comparison to their peers Li W, Ji X, and Wang Z, scientists Zhang Y and Wang Y have written more publications on this subject.

The three-box graph visually depicts the intricate network of connections among cited references, authors, and author keywords, offering invaluable insights into the role of occludin in the pathogenesis of BBB damage in ischemic stroke spanning the years 2000–2023.

The Sankey diagram (Figure 6) illustrates the connections between various scientific journals, authors, and research topics. The journals represented are *Frontiers in Pharmacology*, *PLOS One*, *Stroke*, *Aging and Disease*, *Molecular Neurobiology*, and *Scientific Reports*. Authors such as Zhang Y, Ji X, Li W, Wang Z, Wang Y, Li Y, Li X, Liu KJ, Zhang X, and Liu X are shown contributing to research areas including the BBB, ischemic stroke, occludin, stroke, tight junction proteins, inflammation, tight junctions, and ischemia.

The article "Bibliometric Analysis of the Role of Occludin in the Pathogenesis of Stroke" was published in 2024. Journal: Oxid Med Cell Longev.

### 3.4. Global Scientific Landscape

Over the span of a decade, China and the USA emerged as leaders in scientific production among countries, contributing 365 and 126 publications, respectively, with Germany following closely with 33 publications, South Korea with 30, and Japan and Switzerland with 15 each (Table 1). In terms of publication patterns, China displayed a pronounced inclination toward single-country productions, constituting 86.2% of its publications. Similarly, the United States exhibited a high rate of single-country publications, accounting for 24.2%. Collaboration strength was predominantly observed in partnerships involving the United States and China.

The global collaboration in research on BBB damage in ischemic stroke is depicted in this map (Figure 7). The countries with the greatest number of published articles on a certain topic are indicated by dark blue color. Leading the way in research on BBB impairment in ischemic stroke are the United States and China. Countries with modest but noteworthy research contributions are indicated by light blue. The degree of collaboration between countries is shown by the thickness of the lines connecting them. More collaborative research between the designated nations is indicated by a thicker line. Important international partnerships in this field are highlighted by the lines that connect the United States and China to other nations. The geographic distribution of scientific resources and interest in the subject is reflected in the primary hubs of collaboration, which are in North America, Europe, and East Asia.

As a result, the map makes it evident which nations are actively investigating how ischemic stroke damages the BBB and how they cooperate to produce scientific findings.

### 3.5. Keyword Trends and Emerging Topics

A chronological analysis of important keywords shows that “Occludin” received a peak citation in 2023. Topics such as “blood–brain barrier” (13%), “occludin” (13%), and “ischemic stroke” (12%) also appear quite frequently, demonstrating a continued interest in understanding the role of proteins in the pathogenesis of strokes (Figure 8(a)).

The prevalent author keywords were scrutinized using Biblioshiny, encompassing frequent terms associated with “occludin,” revealing an upward trend in 2023. The frequencies of keywords like “blood–brain barrier” and “stroke” have demonstrated relative stability over time. Notably, a surge in interest is evident in this domain, as indicated by the substantial number of publications in 2023 (Figure 8(b)).

In essence, this study presents a comprehensive review of global research pertaining to the involvement of occludin in BBB damage during ischemic stroke. Throughout recent decades, the study has identified prominent journals, influential articles, and collaborations among institutions, authors, and countries, while also pinpointing significant and emerging keywords. These findings yield invaluable insights into the research landscape, shedding light on prospective avenues for future investigations (Figure 9).

The article "Bibliometric Analysis of the Role of Occludin in the Pathogenesis of Stroke" was published in 2024. Journal: Oxid Med Cell Longev.

## 4. Discussion

In recent years, the application of bibliometric analysis and scientific mapping has burgeoned, reflecting the growing interest within the scientific community to glean insights from comprehensive bibliometric assessments. This study contributes to this evolving field by employing bibliometric analysis to unravel the intricate landscape of occludin research in the context of BBB damage during ischemic stroke. The significance of bibliometric analysis lies in its ability to elucidate the impact of research fields, identify influential papers, and enhance our understanding of the broader intellectual context within specific domains.

Although research publications on this topic are distributed globally, studies originating from China and the United States constituted a predominant share, encompassing 77.5% of all publications. This dominance likely stems from the pioneering efforts of researchers in these countries, coupled with substantial financial support allocated to this field. Collaboration-wise, China and the United States emerged as frontrunners, jointly producing 25 publications. The bulk of these articles surfaced between 2020 and 2022.

Institutionally, China secured all positions within the top 10 institutions concerning publication volume, underscoring the collaborative endeavors among authors across diverse Chinese institutions. China exhibits global leadership in tight junction protein research related to ischemic stroke not only in terms of publication volume but also in hosting influential research establishments in this domain.

Journal analysis revealed that “Brain Research” and “Scientific Reports” stand among the prominent contributors, both falling within the JCR Q1 subregion with impact factors surpassing 3. Additionally, esteemed neuroscience journals such as the *Journal of Cerebral Blood*, *Stroke*, and *Aging and Disease* have disseminated numerous high-quality research findings, emphasizing the pivotal role of occludin in BBB damage during ischemic stroke. This journal analysis offers valuable guidance for researchers seeking to publish articles in this specific field.

The most highly cited article, titled “Cerebral microvascular changes in permeability and tight junctions induced by hypoxia-reoxygenation,” was published on April 1, 2002, in the journal *Heart and Circulatory Physiology* by the National Institute of Neurological Disorders and Stroke. This article delineates that hypoxia induces heightened paracellular permeability, a phenomenon significantly mitigated by both hypoxic conditions and subsequent reoxygenation. It elucidates the impact of these conditions on the expression of tight junction proteins, notably occludin, within the brain's microvasculature during ischemic stroke [16].

The article "Bibliometric Analysis of the Role of Occludin in the Pathogenesis of Stroke" was published in 2024. Journal: Oxid Med Cell Longev.

The second most cited article titled “Matrix metalloproteinase-2-mediated occludin degradation and caveolin-1-mediated claudin-5 redistribution contribute to BBB damage in the early stage of ischemic stroke” was published in *The Journal of Neuroscience*. Conducted by Liu et al. [17] from the Department of Medical Microbiology and Immunology at the University of South China School of Medicine, the study uncovered the depletion of occludin protein and the redistribution of claudin-5 within ischemic brain microvessels. These findings underscore that cerebral ischemia triggers two concurrent processes: MMP-2-mediated occludin degradation and claudin-5 redistribution, both leading to early disruption of the BBB, particularly relevant when employing thrombolysis during stroke treatment [17].

The most prolific researcher in investigating occludin's role in BBB damage is Zhang Y from the Department of Neurosurgery at Shenzhen Second People's Hospital in Shenzhen, China, with a publication record of 15 papers. The most frequently cited article (cited 44 times), titled “Occludin degradation makes brain microvascular endothelial cells more vulnerable to reperfusion injury in vitro,” was published in the *Journal of Neurochemistry* in February 2021. This paper delineates that heightened dietary sodium intake exacerbates BBB dysfunction following ischemic brain injury. Furthermore, the worsening of BBB damage potentially results from the inhibitory effects of sodium on ZO-1 and occludin proteins associated with endothelial tight junctions [18].

The second most cited article authored by scientist Zhang Y, with 43 citations, is titled “Nomilin protects against cerebral ischemia-reperfusion-induced neurological deficits and blood-brain barrier disruption via the Nrf2 pathway.” This publication showcases how nomilin effectively alleviates oxidative stress and facilitates the expression of erythroid 2-related factor 2 (Nrf2). These findings strongly suggest that the depletion of tight junction proteins within the microvasculature is plausibly mediated by oxidative stress [19].

The third most cited article, with 27 citations, is titled “Occludin degradation makes brain microvascular endothelial cells more vulnerable to reperfusion injury in vitro.” This paper investigates the premise that occludin degradation in brain microvascular endothelial cells, triggered by cerebral ischemia, heightens their susceptibility to stress stimuli. Consequently, this renders the cells more prone to endothelial damage, thereby exacerbating their progression toward cell death. The study utilized an in vitro model of oxygen–glucose deprivation (OGD) to simulate conditions of cerebral ischemia. Results revealed that OGD-induced occludin degradation or the deliberate reduction of occludin expression could escalate brain microvascular endothelial cell demise, encompassing apoptosis and pyroptosis, during the subsequent reoxygenation phase [20].

The article "Bibliometric Analysis of the Role of Occludin in the Pathogenesis of Stroke" was published in 2024. Journal: Oxid Med Cell Longev.

A substantial portion of the research received funding through grants provided by the National Natural Science Foundation of China (81070943) [18, 20, 21, 22, 23, 24, 25, 26]. The second most cited author, Wang Y, affiliated with the Department of Neurology at Huazhong University of Science and Technology in Wuhan, China, authored the most cited article (79 times) titled “Recombinant Human Sonic Hedgehog Protein Regulates the Expression of ZO-1 and Occludin by Activating Angiopoietin-1 in Stroke Damage,” published in July 2013. The study revealed a significant increase in angiopoietin-1 protein levels in the culture medium of astrocytes treated with Sonic Hedgehog. Moreover, Sonic Hedgehog notably elevated the expression of zonula occludens-1 (ZO-1), occludin, and angiopoietin-1 in brain microvessel endothelial cells. Remarkably, the inhibition of Sonic Hedgehog's effects on the expression of ZO-1 and occludin was observed with cyclopamine and an angiopoietin-1 neutralizing antibody, respectively [27].

These findings suggest that in the context of ischemic strokes, Sonic Hedgehog primarily stimulates the production of angiopoietin-1 in astrocytes. Subsequently, the secreted angiopoietin-1 acts on brain microvessel endothelial cells, triggering the activation of ZO-1 and occludin. This activation contributes to the restoration of tight junctions, leading to a reduction in brain edema and mitigating BBB permeability [27]. A substantial portion of the research was also supported by grants from the National Natural Science Foundation of China (81070943) [27, 28, 29, 30, 31, 32].

The keywords within a scientific article serve as a reflection of the overarching research themes, thereby offering valuable insights into significant topics and leading directions within a specific field of study. Analyzing the frequency and co-occurrence of keywords aids in identifying pivotal areas of focus. Based on the outcomes derived from the cluster analysis of keywords, the subsequent recommendations are proposed for future investigations concerning the role of occludin in BBB damage during ischemic stroke. The ischemic stroke event involves the engagement of nearly all types of brain cells, underscoring the comprehensive impact on brain physiology. The conceptual framework of the “neurovascular unit” has been instrumental in enhancing our comprehension of central nervous system pathologies, notably stroke. Mounting evidence signifies that BBB disruption correlates with occludin and claudin-5 degradation in brain tissue, as well as the presence of occludin in the bloodstream following a stroke episode.

The article "Bibliometric Analysis of the Role of Occludin in the Pathogenesis of Stroke" was published in 2024. Journal: Oxid Med Cell Longev.

Consequently, delving into the potential role of occludin within neurovascular units—encompassing neurons, astrocytes, and microglial cells—and its interplay with tight junction proteins governing BBB integrity stands as a pivotal and clinically significant pursuit in understanding ischemic stroke pathology [33].

The current study faces several limitations that warrant acknowledgment. Primarily, the utilization of solely the Scopus database for literature search might lead to the exclusion of certain relevant publications, potentially resulting in an underestimation of citations. Consequently, this may not wholly capture the entirety of studies focusing on occludin's role in BBB damage during ischemic stroke.

Second, the Bibliometrix software employed lacks the capability to discern between first and corresponding authors, as well as authors sharing the same name but associated with different departments. This limitation could affect the accuracy of author-related analyses.

Lastly, the existing Bibliometrix software exhibits constraints in setting standardized parameters, thereby predisposing the software clustering process to partial data loss. This inherent limitation might yield unexpectedly divergent analysis outcomes.

Given these limitations, it is essential to acknowledge the need for further refinement in designing bibliometric analyses to address these shortcomings. Enhancements in methodological approaches are necessary to ensure more comprehensive and precise assessments in studies like this one.

### 4.1. Limitations

While this study provides a comprehensive overview of occludin research in ischemic stroke, certain limitations merit acknowledgment. The analysis is contingent on the available literature within the Web of Science and Scopus databases, potentially omitting relevant publications from other sources. Additionally, the bibliometric approach relies on the accuracy and consistency of the metadata within the databases, introducing a degree of dependence on the quality of indexing and categorization. If significant scientific discoveries are published in less prestigious publications, they could not receive the recognition they deserve. To get a more thorough research assessment, it is advised to diversify assessment indicators by integrating several indicators and assessment techniques, such as expert consultation, peer review, and qualitative analysis. Furthermore, it is possible that biases related to language and geography prevented non-English speaking nations' scientific contributions from being acknowledged.

The article "Bibliometric Analysis of the Role of Occludin in the Pathogenesis of Stroke" was published in 2024. Journal: Oxid Med Cell Longev.

### 4.2. Strengths of the Study

The strength of this study lies in its systematic bibliometric approach, encompassing a wide range of sources to provide a holistic view of occludin research in ischemic stroke. The analysis spans a substantial period, capturing trends and developments over time. The incorporation of multiple parameters, including authorship, citations, and keyword analysis, enriches the understanding of the research landscape and offers valuable insights for future investigations. The identification of key journals, prolific authors, and influential keywords provides a foundation for researchers and policymakers to navigate the evolving field of occludin research in stroke pathogenesis.

## 5. Conclusion

The past decade has witnessed a significant surge in research focused on tight junction proteins and their implications in BBB damage associated with ischemic stroke. This growth is reflected in the substantial contributions from China and the United States, with these nations prominently represented among the authors at the forefront of this field. Within this intricate network, occludin, a key tight junction protein, has emerged as a linchpin in regulating BBB integrity and permeability.

In the specific context of ischemic stroke, the consequential BBB damage is intricately linked to hemorrhagic transformation. Notably, our analysis positions occludin as a potential biomarker with significant promise for the early diagnosis of hemorrhagic transformation in ischemic stroke. The recognition of occludin's pivotal role not only expands our understanding of the molecular mechanisms underpinning stroke pathogenesis but also introduces a potential avenue for clinical applications in the realm of stroke diagnostics.

The insights gleaned from this literature analysis not only highlight the current state of research but also underscore the imperative for more extensive exploration into tight junction proteins, encompassing occludin and claudin-5, particularly in the context of acute cerebral ischemia. The identified knowledge gaps and emerging trends, especially relevant to the unique healthcare landscape in Kazakhstan, emphasize the necessity for further scientific research in this region.

The article "Bibliometric Analysis of the Role of Occludin in the Pathogenesis of Stroke" was published in 2024. Journal: Oxid Med Cell Longev.

Moving forward, continued efforts in elucidating the intricate dynamics of tight junction proteins, including occludin, hold the potential to refine our understanding of BBB regulation in ischemic stroke. This knowledge, in turn, may pave the way for the development of targeted therapeutic interventions and diagnostic strategies, offering tangible benefits to stroke patients worldwide. The culmination of these efforts will not only contribute to the scientific discourse but also carry profound implications for the clinical management and outcomes of ischemic stroke, marking a significant stride toward enhancing global stroke care.

## Figures and Tables

**Figure 1:** The flowchart of the screening process using PRISMA to perform bibliometric analysis of the role of occludin in the pathogenesis of stroke.

**Figure 2:** Number of published articles by year to show the role of occludin in the pathogenesis of stroke.

**Figure 3:** The plot of Broadford's law identified 12 core journals on the role of occludin in the pathogenesis of stroke.

**Figure 4:** Most frequently published journals show the role of occludin in the pathogenesis of stroke.

**Figure 5:** Most frequently published authors show the role of occludin in the pathogenesis of stroke.

**Figure 6:** Three-field plot representing inflows and outflows among cited references, authors, and author keywords on the role of occludin in the pathogenesis of blood–brain barrier damage in ischemic stroke from 2000 to 2023. *Abbreviations*. SO, source; AU, authors; and DE; keywords.

**Figure 7:** Map of global collaboration on blood–brain barrier damage in ischemic stroke. The intensity of color saturation corresponds to the increasing number of articles within each country. The collaboration between countries is depicted through the thickness.

**Figure 8:** TreeMap (a) and scatterplot (b) representing the author's top 10 keywords in the study of occludin in the pathogenesis of ischemic stroke (2000–2023).

**Figure 9:** The timeline of the trend topics. Each bubble indicates the peak of frequency used for each, while the line indicates the years it was used.

**Table 1:** Leading publishing countries on damage to the blood–brain barrier in ischemic stroke (2000–2023).

Country	Number of articles
China	365
USA	126
Germany	33
South Korea	30
Japan	15
Switzerland	15
Poland	12
France	10
UK	8
Italy	6

## Data Availability

All data generated or analyzed in this study can be obtained from the corresponding author upon request.
